This article has been retracted.

# Downgrading MELD Improves the Outcomes after Liver Transplantation in Patients with Acute-on-Chronic Hepatitis B Liver Failure

**DOI:** 10.1371/journal.pone.0030322

**Published:** 2012-01-24

**Authors:** Qi Ling, Xiao Xu, Qiang Wei, Xiaoli Liu, Haijun Guo, Li Zhuang, Jiajia Chen, Qi Xia, Haiyang Xie, Jian Wu, Shusen Zheng, Lanjuan Li

**Affiliations:** 1 Key Lab of Combined Multi-Organ Transplantation, Ministry of Public Health, Division of Hepatobiliary and Pancreatic Surgery, Department of Surgery, First Affiliated Hospital, Zhejiang University School of Medicine, Hangzhou, Zhejiang, China; 2 State Key Lab for Diagnosis and Treatment of Infectious Diseases, Department of Infectious Diseases, First Affiliated Hospital, Zhejiang University School of Medicine, Hangzhou, Zhejiang, China; Copenhagen University Hospital Gentofte, Denmark

## Abstract

**Background:**

High score of model for end-stage liver diseases (MELD) before liver transplantation (LT) indicates poor prognosis. Artificial liver support system (ALSS) has been proved to effectively improve liver and kidney functions, and thus reduce the MELD score. We aim to evaluate whether downgrading MELD score could improve patient survival after LT.

**Methodology/Principal Findings:**

One hundred and twenty-six LT candidates with acute-on-chronic hepatitis B liver failure and MELD score ≥30 were included in this prospective study. Of the 126 patients, 42 received emergency LT within 72 h (ELT group) and the other 84 were given ALSS as salvage treatment. Of the 84 patients, 33 were found to have reduced MELD score (<30) on the day of LT (DGM group), 51 underwent LT with persistent high MELD score (N-DGM group). The median waiting time for a donor was 10 for DGM group and 9.5 days for N-DGM group. In N-DGM group there is a significantly higher overall mortality (43.1%) than that in ELT group (16.7%) and DGM group (15.2%). N-DGM (vs. ECT and DGM) was the only independent risk factor of overall mortality (*P* = 0.003). Age >40 years and the interval from last ALSS to LT >48 h were independent negative influence factors of downgrading MELD.

**Conclusions/Significance:**

Downgrading MELD for liver transplant candidates with MELD score ≥30 was effective in improving patient prognosis. An appropriate ALSS treatment within 48 h prior to LT is potentially beneficial.

## Introduction

One-third of global individuals infected with hepatitis B virus (HBV) reside in China, with 130 million carriers, 30 million chronically infected, and 300 thousand per year HBV-related deaths [1]–[3]. Because of the high prevalence of hepatitis B, acute exacerbation of chronic hepatitis B and acute deterioration of cirrhosis are the most common causes of liver failure, contributing to especially high mortality in China. Most recently, these types of liver failure has been considered as acute-on-chronic liver failure (ACLF), which was clearly defined by Asian Pacific Association for the Study of the Liver as ‘acute hepatic insult manifesting as jaundice and coagulopathy, complicated within 4 weeks by ascites and/or encephalopathy in a patient with previously diagnosed or undiagnosed chronic liver disease’ [4]. When ACLF progresses to multi-organ dysfunction such as hepatorenal syndrome and hepatic encephalopathy, the prognosis is dismal unless liver transplantation (LT), the only definitive therapy to salvage these patients, is performed [4]. Since model for end-stage liver diseases (MELD) score was used for organ allocation, candidates with ACLF have the priority to gain the donor liver and receive emergency LT because patients with ACLF usually have high MELD score [5], [6]. However, ‘high-grade’ (≥30) MELD scores in ACLF indicate poorer prognosis after liver support treatment even LT [6]–[8]. For ACLF patients with MELD score≥30, the 30-day survival was less than 10% after ALSS salvage [7], and the 1-year survival after LT was much lower than that of patients with MELD score <30 (33.3% vs. 77.8%) [9]. Thus when the MELD score is <30 it may be the optimal time to perform LT for patients with ACLF [9].

Artificial liver support system (ALSS) has been proved to be an effective way to improve liver function and thus serve as a bridge to LT [10]. After such treatment, total bilirubin, international normalized ratio, encephalopathy, and serum creatinine can be remarkably improved and thus MELD score was reduced [11]. According to the treatment guidelines for ALSS formulated by Artificial Liver Group, Chinese Association of Infectious and Parasitic Diseases and Chinese Medical Association [12], the management of ACLF patients were principally supportive with ALSS treatment prior to LT. In this study, we performed ALSS to salvage ACLF patients with ‘high-grade’ MELD score. We aim to evaluate whether downgrading pre-transplant MELD score could improve patient survival after LT, and to determine the possible influence factors of downgrading MELD.

## Methods

### Patient characteristics

A total of 189 adult patients with acute-on-chronic hepatitis B liver failure (ACLF-HBV) underwent primary LT between January 2001 and June 2010 at the First Affiliated Hospital, Zhejiang University School of Medicine, China. Informed consent was obtained from all donors and recipients before LT. Each organ donation or transplant in our centre was strictly selected according to the guidelines of the Ethical Committee of our hospital, the regulation of Organ Transplant Committee of Zhejiang province and the Declaration of Helsinki. Of the 189 liver transplant candidates, 126 (113 male and 13 female) representing MELD score ≥30 in the waiting list were enrolled in this prospective study. The study protocol was approved by the Ethics Committee, and written informed consent was obtained from all study patients. Recipients with liver cancer were excluded from the study population. Patient characteristics were summarized in **Table S1**.

All patients received lamivudine combined with low-dose intramuscular hepatitis B immunoglobulin therapy according to our anti-virus protocol [13]. All patients were given standard medical treatments including energy supplements, intravenous infusion of albumin and plasma, and preventive treatment of complications. Of the 126 patients, 42 gained prompt donor livers and received emergency LT without any prior treatment (ELT group), the other 84 were given ALSS treatment before LT. The 84 patients were further divided into two sub-groups according to the MELD score on the day of transplant: decreased MELD group (DGM group, n = 33) (MELD score decreased to a level of <30) and non-decreased MELD group (N-DGM group, n = 51) (persistent high MELD score ≥30).

There are indications for ACLF patients receiving ALSS treatment according to Artificial Liver Group, Chinese Association of Infectious and Parasitic Diseases and Chinese Medical Association [12]. The methods of ALSS included plasma exchange with or without continuous hemodiafiltration or plasma perfusion, and molecular adsorbents recirculating system, as described previously [14]. The specialists from Infectious Diseases Department chose therapies and carried out ALSS treatment 1–3 times per week based on the condition of patients and the facility (availability of plasma or machine). The decision to initiate hemodiafiltration were made by consultant nephrologists to prevent uremia or immediate death from the adverse complications of renal failure [15]. In principle, patients with coagulopathy were indicated for plasma exchange (PE); patients with hepatic encephalopathy were given PE plus plasma perfusion or continuous hemodiafiltration. For patients complicated with hepatorenal syndrome or water – electrolytes imbalance, we applied PE plus continuous hemodiafiltration or molecular adsorbents recirculating system. In DGM group, 106 sessions of ALSS were applied to 33 patients with PE 61 times, PE plus plasma perfusion 21 times, PE plus continuous hemodiafiltration 14 times and molecular adsorbents recirculating system 10 times. In N-DGM group, 149 sessions of ALSS were applied to 51 patients, with PE 69 times, PE plus plasma perfusion 39 times, PE plus continuous hemodiafiltration 20 times and molecular adsorbents recirculating system 21 times. Emergency LT was performed within 72 h after patients became LT candidates for the purpose of our protocol [16].

United Network for Organ Sharing status was used to stratify the patients on the waiting list and allocate donor organs before December 2002, and then substituted by MELD score after January 2003. Post-reperfusion liver biopsies were obtained after liver implantation for histological evaluation of donor liver steatosis. According to the grade of macrovesicular steatosis, liver grafts were categorized into four groups: no steatosis, mild steatosis (<30%), moderate steatosis (30–60%), and severe steatosis (>60%) [17]. Deceased donor liver transplantation (DDLT) and living donor liver transplantation (LDLT) were performed in 93 and 33 cases, respectively. Of 93 donations after cardiac death, 3 were controlled and 90 were uncontrolled. Operation techniques of both DDLT and LDLT were described previously [18], [19]. The primary immunosuppressive regimen was triple therapy incorporating tacrolimus or cyclosporine, mycophenolate and steroid [20]. An IL-2 receptor blocker was used in selected patients.

### Data collection

All patients were followed up closely in the outpatient clinic and data were collected for analysis. Pre-transplant data included age, gender, underlying liver disease, complications, MELD score, serum potassium and sodium, need for ALSS, and need for intensive care. Post-transplant complications, organ function and patient survival were also collected.

MELD was calculated according to the UNOS formula: MELD = 3.78×ln (bilirubin [mg/dl])+9.57×ln (creatinine [mg/dl])+11.20×ln (international normalized ratio)+6.43 and the range of the MELD score is 6–40 [21]. Delta-MELD = MELD score calculated on the day of transplant−MELD score calculated when patients were listed as LT candidates. The post-transplant model for predicting mortality (PMPM) score was calculated at 24 h following transplantation: PMPM score = −5.359+1.988×ln (serum creatinine [mg/dl])+1.089×ln (total bilirubin [mg/dl]) [22].

According to Asian Pacific Association for the Study of the Liver, ACLF was defined as ‘acute hepatic insult manifesting as jaundice (serum bilirubin >5 mg/dl) and coagulopathy (international normalized ratio >1.5 or prothrombin time activity <40%), complicated within 4 weeks by ascites and/or encephalopathy in a patient with previously diagnosed or undiagnosed chronic liver disease’ [4]. The diagnosis of acute exacerbation of chronic hepatitis B was based on findings of fibrous bands and ductular proliferation using by biopsy [4]. The diagnosis of cirrhosis with acute deterioration was based on the presence of hepatocyte necrosis and features of acute hepatitis under the background of cirrhosis [4]. The diagnostic criteria for hepatorenal syndrome was based on the International Ascites Club consensus [23]. The diagnosis of hepatic encephalopathy was based on the clinical manifestations and the signs of brain edema. The severity of hepatic encephalopathy was evaluated by the criteria for grading mental status [14]. Early allograft dysfunction was defined by the presence of at least one of the following characteristics: total bilirubin >10 mg/dl, prothrombin time ≥17 s and hepatic encephalopathy from days 2 to 7 post-transplantation [24]. Acute kidney injury was defined as an elevated level of serum creatinine (>1.5 mg/dL) or/and need for hemodiafiltration during the first post-transplant week [25]. Acute rejection was diagnosed routinely in liver biopsies according to the Rejection Activity Index criteria. Bacterial and fungus infection was diagnosed on the basis of primary culture, while viral infection was diagnosed on the basis of PCR result in the blood sample. Biliary complications were classified as bile leakage and stenosis. Bile leakage was primarily diagnosed on the basis of bilirubin in abdominal drainage, newly inserted pigtail, or cholangiography. Biliary stenosis was diagnosed on the basis of an overt dilatation of the intra-hepatic duct according to the imaging findings.

### Statistical methodology

The Kolmogorov-Smirnov test was used to evaluate normality. Quantitative variables were presented as mean ± SD. Categorical variables were expressed as values and percentages. Student's *t* test or Mann-Whitney test was used to compare quantitative variables, while Chi-square test was used to compare categorical variables. Kaplan-Meier method with log-rank test and COX regression analysis were used for survival analysis. Logistic regression analysis was used for influence factors analysis. Variables with statistically significance in univariate analysis were taken for a forward stepwise multivariate analysis. SPSS for Windows version 11.0 (SPSS Inc., Chicago, IL) was used to complete all the analyses, and a *P* value of <0.05 was considered statistically significant.

## Results

### Pre-transplant ALSS treatment

The liver and kidney functions were improved temporarily after each ALSS session in all treated patients, presenting a significantly decreases in total bilirubin (33.4±12.7 mg/dL vs. 16.3±9.7 mg/dL, *P*<0.001), alanine aminotransferase (169±135 U/L vs. 78±67 U/L, *P* = 0.012), aspartate aminotransferase (202±107 U/L vs. 101±80 U/L, *P*<0.001), prothrombin time (32.6±10.3 s vs. 21.5±6.4 s, *P* = 0.024), international normalized ratio (3.36±0.95 vs. 2.17±0.76, *P* = 0.018) and serum creatinine (2.04±1.04 mg/dL vs. 1.21±0.83 mg/dL, *P* = 0.041). However, after all sessions of ALSS treatment, DGM group showed better liver and kidney functions than N-DGM group (**Table 1**).

**Table 1:** Changes of biochemistry parameters after all sessions of ALSS treatment.

	DGM group	N-DGM group
	(n = 33)	(n = 51)
Total bilirubin		
On the day of listing	28.4±11.8	26.6±10.2
On the day of transplant*	19.6±8.6	29.2±12.4
Alanine aminotransferase		
On the day of listing	132±123	148±102
On the day of transplant*	67±46	169±97
Aspartate aminotransferase		
On the day of listing	195±112	202±96
On the day of transplant*	98±76	213±105
Prothrombin time		
On the day of listing	28.4±11.2	30.1±10.6
On the day of transplant*	20.2±7.3	31.2±9.8
International normalized ratio		
On the day of listing	2.8±0.9	2.9±1.1
On the day of transplant*	2.1±0.7	3.0±1.2
Serum creatinine		
On the day of listing	1.2±0.6	1.5±1.0
On the day of transplant*	1.1±0.7	1.7±1.1

Abbreviations: ALSS, artificial liver support system; DGM, downgraded MELD; MELD, model for end-stage liver disease; N-DGM, non-downgraded MELD;

*: N-DGM group vs. DGM group, *P*<0.05;

Complications which occurred in 31 patients (24.6%) during ALSS therapy included skin rash (11.1%), hypotension (6.3%), blood coagulation in perfusion cartridges (3.2%), local bleeding (3.2%) and infection (2.4%).

The median interval time from the last ALSS treatment to LT was 48 h (range: 24 h–8 d) in DGM group and 72 h (24 h–25 d) in N-DGM group (*P* = 0.147). The median waiting time for a donor liver was 10 days (range: 4–43 d) in DGM group and 9.5 days (range: 4–70 d) in N-DGM group, (*P* = 0.792).All recipients and donors experienced uneventful operative procedure.

### Post-transplant complications

The incidence of post-transplant hemorrhage, early allograft dysfunction, acute kidney injury, acute rejection, infection and biliary complication was 10.3%, 28.6%, 15.9%, 12.7%, 29.4% and 13.5%, respectively. Most of complications (82.4%) developed in the first post-transplant month. In N-DGM group there was a significantly higher prevalence of acute kidney injury than that in ELT group (39.2% vs. 14.3%, *P* = 0.008) and DGM group (39.2% vs. 9.1%, *P* = 0.002), and higher incidence of infection than that in ELT group (43.1% vs. 19.0%, *P* = 0.013) and DGM group (43.1% vs. 21.2%, *P* = 0.039).

### Patient survival

Of all 126 patients, 34 passed away during a median of 1.53 (0.03–9.86) years follow-up (**Figure 1**). The 1-month, 1-year and 5-year mortality was 16.7%, 24.6% and 27.0%, respectively, in the whole study population. There was a significantly higher overall mortality in N-DGM group than that in ELT group (43.1% vs. 16.7%, *P* = 0.007) and DGM group (43.1% vs. 15.2%, *P* = 0.006).

**Figure 1:** Outcomes of all 126 ACLF patients with pre-transplant MELD ≥30. ALSS, artificial liver support system; DGM, downgraded MELD; ELT, emergency liver transplantation; GVHD, graft versus host disease; MELD, model for end-stage liver disease; MODS, multi-organ dysfunction syndrome; N-DGM, non-downgraded MELD.

Most of deaths (21/34) occurred during the first post-transplant month. The causes of early death (<30 d) were multi-organ dysfunction syndrome (MODS, n = 15), hemorrhage (n = 4) and infection (n = 2). The early mortality was 14.3%, 9.1%, and 23.5% in the ELT group, DGM group and N-DGM group, respectively.

Patient cumulative survivals were presented in **Figure 2** and did not differ significantly between patients undergoing LDLT and those receiving DDLT (*P* = 0.338), patients with acute exacerbation of chronic hepatitis B and those with acute deterioration of cirrhosis (*P* = 0.655), or DGM group and ELT group (*P* = 0.901). There was a significantly lower patient cumulative survival in N-DGM group than that in NDM group (*P* = 0.008) and ELT group (*P* = 0.006). Patients with PMPM score <−1.4 had a remarkably higher cumulative survival than those with PMPM score >−1.4 (*P*<0.001).

**Figure 2:** Comparison of patient cumulative survivals. Kaplan-Meier analysis was used to compare survivals between patients underwent LDLT and those received DDLT (A), patients with acute exacerbation of chronic hepatitis B and those with acute deterioration of cirrhosis (B), ELT group, DGM group and N-DGM group (C), patients with PMPM score <−1.4 and those with PMPM score >−1.4 (D). LDLT, living donor liver transplantation; DDLT, deceased donor liver transplantation; ELT, emergency liver transplantation; DGM, downgraded MELD; N-DGM, non-downgraded MELD; PMPM, post-transplant model for predicting mortality.

### Risk factors of death

Univariable analysis showed the following pre-transplant factors that were significantly related to the early death (<30 d): N-DGM (vs. ECT and DGM), delta-MELD, hepatorenal syndrome, infection, and serum sodium. These factors were then entered into the multivariable COX analysis and the independent risk factors of early death were N-DGM (vs. ECT and DGM) (RR = 2.426, *P* = 0.049) and hepatorenal syndrome (RR = 2.422, *P* = 0.039) (**Table 2**).

**Table 2:** COX regression for pre-transplant influence factors of patient death.

	Univariable analysis		Multivariable analysis	
	Risk ratio (95% CI)	*P*	Risk ratio (95% CI)	*P*
Early mortality (<30 d)				
N-DGM (vs. ECT and DGM)	3.112 (1.331–7.273)	0.009	2.426 (1.002–5.881)	0.049
Delta-MELD	1.086 (1.006–1.173)	0.035		
Hepatorenal syndrome	3.136 (1.404–7.005)	0.005	2.422 (1.047–5.600)	0.039
Infection	2.372 (1.065–5.281)	0.034		
Serum sodium	0.927 (0.875–0.981)	0.008		
Overall mortality				
N-DGM (vs. ECT and DGM)	3.196 (1.623–6.294)	0.001	3.209 (1.499–6.869)	0.003
Delta-MELD	1.083 (1.018–1.152)	0.011		
Hepatorenal syndrome	2.015 (1.050–3.867)	0.035		
Serum sodium	0.938 (0.895–0.984)	0.009		

Abbreviations: CI, confidence interval; DGM, downgraded MELD; ELT, emergency liver transplantation; MELD, model for end-stage liver disease; N-DGM, non-downgraded MELD.

N-DGM (vs. ECT and DGM), delta-MELD, hepatorenal syndrome and serum sodium were found significantly associated with overall death, however, only N-DGM (vs. ECT and DGM) (RR = 3.209, *P* = 0.003) was the independent risk factor of overall death (**Table 2**).

### Influence factors of downgrading MELD

Compared with DGM group, N-DGM group showed older age, more hepatic encephalopathy, more hepatorenal syndrome, and more infection (**Table 3**). Logistic regression univariable analysis demonstrated age >40 y, hepatic encephalopathy, hepatorenal syndrome, infection and the interval from last ALSS to LT >48 h were negative influence factors of downgrading MELD. Then these factors were entered into multivariable analysis and the independent negative factors influencing the reduction of MELD were age >40 y (OR = 0.240, *P* = 0.015) and the interval from last ALSS to LT >48 h (OR = 0.261, *P* = 0.022).

**Table 3:** Logistic regression for influence factors of downgrading MELD.

	Univariable analysis		Multivariable analysis	
	Odds ratio (95% CI)	*P*	Odds ratio (95% CI)	*P*
Age >40 y (vs. ≤40 y)	0.292 (0.112–0.759)	0.012	0.240 (0.076–0.760)	0.015
Hepatic encephalopathy (yes vs. no)	0.400 (0.162–0.986)	0.047		
Hepatorenal syndrome (yes vs. no)	0.250 (0.088–0.708)	0.009		
Infection (yes vs. no)	0.250 (0.088–0.708)	0.009		
Interval from last ALSS to LT >48 h (vs. ≤48 h)	0.307 (0.106–0.888)	0.029	0.261 (0.083–0.824)	0.022

Abbreviations: ALSS, artificial liver support system; CI, confidence interval; MELD, model for end-stage liver disease; LT, liver transplantation.

## Discussion

There is a lack of a clear definition of ACLF until the Asian Pacific Association for the Study of the Liver consensus meeting in 2009. In China, where there is particularly high prevalence of hepatitis B and huge population of hepatitis B patients, ACLF has long been considered as a kind of severe viral hepatitis according to the Viral Hepatitis Protection and Cure Guideline established by the Chinese Infection and Hepatology Association. Although ACLF is believed to be reversible, the reversibility depends on the severity and nature of the acute insulting and the degree of underlying chronic liver disease [4]. For ACLF-HBV patients with ‘high-grade’ MELD score (≥30), resolving liver failure and sustaining life can be hardly achieved [7]. Recent Studies demonstrated extremely high short-term mortality of >90% in ACLF patients with MELD scores ≥30 under conventional medications [7], [8]. ALSS treatment could slightly decrease the mortality (68–91%) and therefore serve as a bridge to LT [7], [8]. Thus LT was considered as the only curative therapy for these patients. Since MELD score has been widely used for donor organs allocation, ACLF patients usually have the priority to gain a donor liver and receive emergency LT, which can effectively resolve endotoxemia and liver failure before ACLF greatly progresses [26]. As a result, the short-term and long-term survivals were satisfactory for ACLF patients receiving emergency LT. This indicated that LT should be considered as the first-line treatment option in these patients. But timely LT is not always available because of the donor shortage. The acute loss of liver function on the basis of chronic hepatitis or cirrhosis can dramatically accumulate massive metabolic toxins, leading to organ impairment and then causing severe complications such as infection and organ failure [4], [27]. Therefore, we performed ALSS as a salvage treatment in all study patients who had no chance to receive emergency LT as recommended by Artificial Liver Group, Chinese Association of Infectious and Parasitic Diseases and Chinese Medical Association.

For patients receiving ALSS treatment prior to LT, only those with decreased MELD score showed encouraging long-term survival after LT. Persistently high MELD score before LT was identified as the major independent risk factor of both early death and overall death. ALSS could create good environment for the self-regeneration of remained hepatocytes and thus led to great amelioration in encephalopathy, total bilirubin, international normalized ratio and creatinine, as well as a decrease in MELD score [11], [14]. In this sense, pre-transplant salvage treatment could be considered as ‘valid’ and ‘invalid’ in patients with decreased MELD and non-decreased MELD, respectively. For patients with non-reduced MELD, high levels of circulating endotoxins could be even elevated throughout the transplantation procedure and during the early post-transplant period, and then contribute to high morbidity and mortality [28]. For patients with decreased MELD, ALSS treatment improved patient conditions and enhanced the surgical tolerance. Although their waiting time was much longer than patients receiving emergency LT, patients experienced uneventful procedure during peri-operative period and showed comparable incidence of post-transplant complications and low early mortality. Since a reduced MELD score played a crucial role in the patient outcome, further identification of the potential influence factors of downgrading MELD was essential.

Age, hepatic encephalopathy, hepatorenal syndrome, infection and treatment interval (from last ALSS to LT) were found to be associated with reduction of MELD score. The cut-off values of age and treatment interval were chosen according to the clinical experience. Old age has been considered as a risk factor of patient prognosis after LT especially in patient with liver failure [29]. However, the impact of old age on the efficacy of ALSS has been rarely studied and need clarification in the further research. As well known, ALSS could only substitute a few elementary liver functions but not replace the entire spectrum of hepatic function. It is beneficial to ameliorate the microenvironment of the liver, but the function recovery is basically dependent on the self-regeneration of remained hepatocytes. In this study, hepatic encephalopathy, hepatorenal syndrome and infection, which reflected clinical severity of end-stage liver disease, were not independent influence factors. Consequently, the ability of ALSS to improve the MELD score might not be determined by the severity of underlying diseases. For ACLF patients with ‘high-grade’ MELD scores, whose livers have virtually little chance of self-regeneration [7], our results revealed the efficacy of ALSS was more likely determined by the therapeutic timing. The multivariate analysis showed long treatment interval (last ALSS to LT >48 h) played central role in the reduction of MELD score. A recent study investigated the dynamic change of total bilirubin, international normalized ratio and creatinine levels after ALSS, showing a significant improvement at 24 h, however, deterioration at 72–120 h post-ALSS [11] in these parameters. Thus many patients received several sessions of ALSS treatment before LT because their conditions deteriorated soon after one session of salvage treatment. These results suggested that consecutive sessions of ALSS were indeed effective in bridging critically ill patients to LT. An appropriate or even additional ALSS treatment within 48 h prior to LT was beneficial for improving patient's condition and downgrading MELD, thus further reducing the post-transplant mortality.

Hepatorenal syndrome was found to be another independent risk factor of early deaths. Hepatorenal syndrome occurs predominantly in advanced cirrhosis and also develops in severe liver failure, and may accompany the worst prognosis among all the complications of cirrhosis. There has been a consensus that pre-transplant renal dysfunction was a strong predictor of poor prognosis after LT, especially in patients with high MELD score [15], [30], [31]. In some LT candidates with severe kidney impairment, renal function maybe deteriorated after LT and combined liver kidney transplantation should be considered [15], [32]. Our results were consistent with the previous studies that high prevalence of hepatorenal syndrome contributed to the high incidence of post-transplant acute kidney injury and high mortality. The findings indicated that management of pre-transplant renal dysfunction was of vital importance for reducing the morbidity and mortality in patients with ACLF.

In the present study, we found several potential influencing factors including the quality of donors, HBV DNA load and cirrhosis background did not affect the patient survival. We have previously reported that moderately steatotic liver grafts provide adequate function in the first phase after transplantation and can be used for transplantation [17]. The shortage of donor organs has required us to use moderately but not severe steatotic liver grafts in order to expand the donor pool. HBV DNA load has been reported to be a predictor of poor prognosis among ACLF patients with high MELD score [8]. However, no good prognostic ability was seen among those critically ill patients after liver transplantation. Since lamivudine combined with low-dose intramuscular hepatitis B immunoglobulin therapy were routinely used in our center, HBV has been well controlled during the peri-operative period and the HBV recurrent rate has largely been reduced [13]. Other prognostic factors rather than HBV DNA load may play key roles in patient survival. Post-transplant model for predicting mortality (PMPM) was proven once again to be a good survival predictor even in this special study population [22]. In our centre, we use PMPM as an alarm bell for early recognition and prediction of poor outcome.

There were several limitations in this study. First, the endotoxin levels were not measured in all study population and thus not included in the data analysis. The comparison of circulating endotoxin levels during the peri-operative period among ELT, DGM and N-DGM groups, and the possible negative effect of high circulating endotoxin level on patient outcomes should be further evaluated in ACLF patients with high MELD score. Second, this study was limited in a Chinese population with severe hepatitis B. These study results should be further verified in a heterogeneous Western population with a relatively low incidence of hepatitis B. Third, this was not a randomized study because the selection of patients for emergency LT had to follow the organ allocation system. Only the critically ill patients received timely ALSS treatment which was limited by the availability of plasma and machine. Therefore, there were several confounding variables which may affect the results. A randomized study between groups that have and do not have prompt ALSS (within 48 h prior to LT) to reduce MELD scores should be conducted to verify our results.

In summary, for ACLF patients with ‘high’ MELD score, emergency LT was the choice and reduction of the MELD score before LT was effective in improving the patient prognosis. An appropriate ALSS treatment within 48 h prior to LT can be beneficial.

## Supporting Information

Table S1 Demographic comparisons among the ELT, DGM and N-DGM groups.
(DOC)
